# Application of an Effective Statistical Technique for an Accurate and Powerful Mining of Quantitative Trait Loci for Rice Aroma Trait

This article has been retracted.

**DOI:** 10.1371/journal.pone.0129069

**Published:** 2015-06-10

**Authors:** Farahnaz Sadat Golestan Hashemi, Mohd Y. Rafii, Mohd Razi Ismail, Mahmud Tengku Muda Mohamed, Harun A. Rahim, Mohammad Abdul Latif, Farzad Aslani

**Affiliations:** 1 Institute of Tropical Agriculture, Universiti Putra Malaysia, 43400 UPM, Serdang, Selangor, Malaysia; 2 Department of Crop Science, Faculty of Agriculture, Universiti Putra Malaysia, 43400, Serdang, Selangor, Malaysia; 3 Bioscience and Agrotechnology Division, Malaysian Nuclear Agency, Bangi, 43000, Kajang, Selangor, Malaysia; 4 Bangladesh Rice Research Institute (BRRI), Gazipur, 1701, Bangladesh; Institute of Cotton Research of Chinese Academy of Agricultural Sciences, CHINA

## Abstract

When a phenotype of interest is associated with an external/internal covariate, covariate inclusion in quantitative trait loci (QTL) analyses can diminish residual variation and subsequently enhance the ability of QTL detection. In the in vitro synthesis of 2-acetyl-1-pyrroline (2AP), the main fragrance compound in rice, the thermal processing during the Maillard-type reaction between proline and carbohydrate reduction produces a roasted, popcorn-like aroma. Hence, for the first time, we included the proline amino acid, an important precursor of 2AP, as a covariate in our QTL mapping analyses to precisely explore the genetic factors affecting natural variation for rice scent. Consequently, two QTLs were traced on chromosomes 4 and 8. They explained from 20% to 49% of the total aroma phenotypic variance. Additionally, by saturating the interval harboring the major QTL using gene-based primers, a putative allele of *fgr* (major genetic determinant of fragrance) was mapped in the QTL on the 8th chromosome in the interval RM223-SCU015RM (1.63 cM). These loci supported previous studies of different accessions. Such QTLs can be widely used by breeders in crop improvement programs and for further fine mapping. Moreover, no previous studies and findings were found on simultaneous assessment of the relationship among 2AP, proline and fragrance QTLs. Therefore, our findings can help further our understanding of the metabolomic and genetic basis of 2AP biosynthesis in aromatic rice.

## Introduction

Scent is considered one of the most important traits of rice grain quality because a strong and pleasant fragrance plays a considerable role in rice marketing [1]. Among more than 100 volatile flavor compounds associated with aromatic rice, 2-acetyl-1-pyrroline (2AP) has been found to be the primary cause of the distinctive aroma in Basmati and Jasmine rice [2]. The key intermediate in the formation of rice flavor, 2AP, is 1-pyrroline formed from proline by Strecker degradation. According to radio-labeling research, the nitrogen contained in the pyrroline ring of proline becomes the nitrogen contained in the pyrroline ring of 2AP in aromatic rice [3]. In fact, 2AP is synthesized by the polyamine pathway and a proline amino acid is a crucial precursor for 2AP [4].

In spite of various genetic and geographic sources of the fragrance trait, QTL mapping, fine mapping, sequence analysis and complementation testing have revealed the *badh2* allele of the *fgr* gene, as the main genetic determinant of aroma in all scented rice lines [5, 6, 7]. The *fgr* gene, located on the 8th chromosome [8, 9, 10], encodes the betaine aldehyde dehydrogenase (BADH) enzyme [11, 12]. In rice, *badh2-E7* [7], with an 8 bp deletion and 3 single nucleotide polymorphisms (SNPs) in the 7th exon [13], and *badh2-E2*, with an identical sequence to the *badh2* allele but involving a 7 bp deletion in the 2nd exon [14], are recessive null alleles for fragrance [15]. Hence, for breeding aromatic rice cultivars, both null alleles can be utilized [14]. However, it has been claimed that *BADH2* is not the only gene governing the scent trait in rice [11, 16, 17].

By various complex statistical procedures, gene number in this quantitative trait has been estimated [8, 18, 19]. However, none of the estimates is completely reliable due to the possibility of genes with minor contributions that are highly affected by environment, in genetic linkage, etc [19]. Regarding this issue, although genetic analyses have always indicated that the aroma trait is governed by recessive monogenic inheritance [20, 21, 22, 23], inconsistent observations in terms of the nature of fragrance inheritance and the number of genetic loci involved [16, 24] have suggested the control by different genes (either dominant or recessive). For instance, the following various modes of aroma inheritance have been reported so far: one main QTL on chromosome 8 and two minor QTLs on chromosomes 3 and 4 [8], two to three recessive or dominant genes [25], two recessive genes [26, 27, 28], one major QTL on chromosome 8 and two minor QTLs on chromosomes 4 and 12 [18], a single dominant gene [17], a dominant suppression epistasis interaction between two genes [29] and an interaction between two genes (complimentary gene action) [29]. Thus, the genetic basis of rice scent has become a controversial and complex issue [5, 15]. However, a very effective technique to cope with such contradictions is inclusion of a covariate (or covariates) in QTL mapping analyses [30] because it might decrease residual variation, increasing the ability to trace QTLs [30]. It is also worth mentioning that this technique can be applied not only to a wide range of traits in plants but also to humans and animals [30]. In addition to find evidence for an additive covariate, it is also of great significance to explore potential QTL *×* covariate interactions [30]. Furthermore, mapping QTLs based on anchor markers, particularly candidate genes that control a favorable trait, can increase the power of QTL detection [31].

Despite the high importance of fragrant rice, few QTL mapping studies for grain 2AP-density have been conducted due to difficult and costly analyses of 2AP [32]. Traditional procedures are less expensive but are subjective and, therefore, not reliable [18]. Thus, for a quantitative and clear assessment of rice scent, 2AP values should be measured using a more sensitive method, such as Gas Chromatography-Mass Spectrometry (GC-MS) [12]. Finally, no molecular research has been performed on the genetic and inheritance basis of flavor in the Malaysian rice gene pool. Hence, this study was undertaken with the aim to accurately discover (i) the genetic inheritance of aroma in a popular Malaysian fragrant rice accession, MRQ74, with an appealing popcorn-like aroma, and (ii) the location and action of the underlying gene(s), using a metabolomic covariate, microsatellites and candidate gene-based sequence polymorphisms, and based on precise measurement of 2AP in rice grains.

## Materials and Methods

### Population Development

‘MR84’, a Malaysian high yielding non-aromatic accession, and ‘MRQ74’, an elite Malaysian aromatic rice cultivar, were obtained from the Malaysian Agriculture Research and Development Institute (MARDI) and used as parental lines in this research. After their hybridization, a single F_1_ plant, a verified hybrid by marker, was self-fertilized to produce F_2_ seeds. Finally, for QTL analysis, 189 of those F_2_ individuals were cultivated in a rice field at Universiti Putra Malaysia (UPM).

### Analytical Quantification of 2-acetyl-1-pyrroline

In order to distinguish fragrant rice kernels from non-fragrant ones and measure 2AP content in F_3_ self-pollinated seeds of each F_2_ line, Gas Chromatography-Mass Spectrometry (GC-MS) (Thermo Scientific, TSQ Quantum XLS, USA) equipped with SPME (Solid-phase microextraction) was used. GC with a TG-5MS capillary column (30 m×0.25μm) and MASS were also used to analyze headspace volatiles (Thermo Scientific, TSQ Quantum XLS, USA). We compared their mass spectra with those in the National Institute of Standards and Technology (NIST, ver. 2.0f, 2008) mass spectral database.

### High-Performance Liquid Chromatography (HPLC) Analysis of Proline

For sample preparation of the rice seeds, 50 μL of extract was removed and dried under vacuum (37°C, 20 mmHg). After, we added and mixed 20 μL of a first coupling reagent, including water, methanol, and triethylamine (TEA) (2:2:1; v/v)]. Then, we dried the sample using a vacuum for 10 min and subsequently reacted it with 30 μL of PITC reagent including methanol, TEA, PITC, and water (7:1:1:1; v/v)] at room temperature for 20 min before drying under a vacuum to remove PITC. Next, the extracted samples were re-dissolved in 500 μL of buffer A, mobile phase for HPLC, and filtered applying a Millipore membrane (0.22 μm). Then, 20 μL of the sample was injected into an HPLC system (model MD-2010; JASCO, Tokyo, Japan) using a gradient system of buffer A (100%-0% after 50 min) and buffer B (0%-100% after 50 min). A C18 reversed-phase column from Alltech (Alltima C18 5U, 250 × 4.6 mm) was used. The operating temperature was adjusted to 43°C. An absorbance of 254 nm was used. The UV absorption spectrum was effective in identification. A standard protein amino acid combination (food hydrolysate A 9656, Sigma) was also prepared.

### DNA Extraction, PCR and Genotyping

We extracted high-quality genomic deoxyribonucleic acid (DNA) from F_2_ leaves for marker screening using a CTAB protocol [33]. For a parental polymorphism assay, 512 pairs of Simple Sequence Repeat (SSR) markers (First BASE Laboratories Sdn Bhd Co., Ltd, Malaysia) and nine gene-based primers were selected from already available rice sequence and genetic linkage maps [34, 35]. These markers were scattered across the entire rice genome. PCR amplification was carried out in a 15-μL reaction mixture containing DNA as the template, 0.1 μM forward and reverse primer, 80 μM dNTPs, 2 mM MgCl2 and 0.5 U of DNA Taq polymerase enzyme. A touchdown PCR protocol from Bradbury et al. [36] was used in which the cycling conditions were an initial denaturation at 94°C for 2 min followed by 30 cycles of 5 s at 94°C, 5 s at 58°C, and 5 s at 72°C and concluded with a final extension at 72°C for 5 min. Then, to resolve the PCR products, 3% MetaPhore gels were used. The particulars of polymorphic markers are shown in S1 and S2 Tables, respectively.

### Data Analysis

The phenotypic data for 2AP and proline content were investigated for normal distribution. Additionally, the standard deviation and mean were calculated. We also examined the deviations from a Mendelian segregation ratio through the Chi-square goodness of fit test. Pearson’s correlation was performed to examine the possible correlation between 2AP and proline values. Subsequently, a scatterplot of phenotypes was created. R statistical software was used for the analyses [37].

Prior to construction of the genetic linkage map, we filtered markers for segregation ratios and genotyping errors. As markers remarkably (*P*< 1e-10) deviated from the expected 1:2:1 ratio in the chi-square test, and a genotyping error LOD = 2 would be excluded from further examination. Polymorphic SSR markers were placed in linkage groups using a minimum 6.0 log of odds (LOD) and a maximum 0.35 recombination frequency. “Plot.rf.” function was used to plot marker order in each group. The final linkage map was created using the “ripple” function (*P* < 0.005). Marker orders conflicting with the physical map were recalculated according to LOD scores. In order to estimate the map distances, Kosambi’s mapping function was used [38]. Accuracy of the linkage map was examined by calculating pair wise resynthesis of fractions across the genome and comparing marker order to the physical location on the rice genome. The R/qtl [39] and RCircos [40] packages were used for linkage analysis and creating a graphical view of entire linkage groups, respectively.

The typical model for interval mapping without considering a covariate is as follows:

$$y_{i}\left|g_{i}\right.\sim N\left(\mu_{gi},\;\right.\left.\sigma^{2}\right)$$

Where:

*y*_*i*_: phenotype

*g*_*i*_: QTL genotype for individual *i*

Based on this model, the residual variation has a normal distribution with constant variance [30]. However, considering an “additive covariate”, denoted *x*, leads to the following model:

$$y_{i}\;=\;\mu \;+\;\beta_{x}x_{i}\;+\;\beta_{g}g_{i}\;+\;\epsilon_{i}$$

The average phenotype is linear in *x*, and the QTL has constant effect, independent of *x*. When there is a quantitative covariate for an inter-cross, there are three parallel regression lines describing the average phenotype as a function of the covariate for individuals with QTL genotypes AA, AB, and BB, respectively [30]. The question is then whether there is a QTL × covariate interaction, which we could investigate by fitting the model with the covariate as strictly additive and then as interactive, and taking the difference in LOD scores; if large, that indicates that there is evidence for a QTL × covariate interaction. Thus, we considered proline as an interacting covariate in our analysis. In the case that *x* is an “interactive covariate”, the model is as follows:

$$y_{i}\;=\;\mu \;+\;\beta_{x}x_{i}\;+\;\beta_{g}g_{i}\;+\;\gamma x_{i}g_{i}\;+\;\epsilon_{i}$$

The coefficient for the QTL *×* covariate interaction, *γ*, shows the difference in the QTL effect among covariate values [30].

Hence, to detect putative genetic areas related to aroma, we used Haley-Knott regression (HK) and included covariate by applying the “addcovar = covar” argument. A “calc.genoprob” function was employed to examine the possibilities of the true underlying genotypes given the observed marker data. To establish statistical significance for the genome scan, significance thresholds were extracted from 1,000 permutations that maintained the relationship between proline and 2AP content and shuffled the relationships between genotypes and phenotypes. Thresholds were based on a genome-wide type I error rate of 5% [30, 41]. Consequently, a LOD score of > 3.3 was utilized to determine QTL for minimizing type II error. Additionally, two-dimensional scans with a two-QTL model were performed with the thresholds according to the findings of 1,000 permutations at a 5% significance level. Subsequently, a multiple QTL mapping approach was employed to identify the true QTLs. For each QTL location, the 95% Bayesian confidence interval was estimated [42]. The additive and dominant impacts and the phenotypic variance percentage explained by each QTL (R^2^) at the maximum LOD score were calculated by the “makeqtl” and “fitqtl” functions. The analyses were performed using R/qtl software [39]. Finally, to name the mapped QTLs, we used a three letter abbreviation for the fragrance trait (frg) followed by the chromosome number on which the QTL was traced [43]. The Cornell SSR map, a genetic linkage map of rice, was used to compare QTL locations identified in the present study.

## Results

### Phenotype and Covariate Performance

In the F_2_ mapping population, the distribution of 2AP measures was between the values of the parental inbred lines without considerable transgressive segregation (Fig 1). Only a part of the F_2_ plants reconstituted the original scent of MRQ74, indicating the action of many genes. For the fragrance characteristics, the Kolmogorov–Smirnov normality test demonstrated that the distribution was not normal (*p* < 0.01) (Mean = 65.9, Std. Deviation = 63.2). The normal curve was skewed towards non-scented parent. The frequency of proline content also had an asymmetric distribution (Mean = 6.7, Std. Deviation = 2.8). Pearson’s correlation revealed a significant correlation between 2AP and proline values (r = 0.6) at the 0.01 level. Additionally, a scatterplot of phenotype versus covariate is shown in Fig 2.

**Fig 1:** Histogram of the 2AP distribution in the F_2_ population developed from MR84 (P_1_) × MRQ74 (P_2_) using quantitative assessment (ppb).

**Fig 2:** Scatterplot of 2AP (ppb) versus proline content (mg/g) for the F_2_ individuals.

### Genotypic Analysis of Mapping Population

In total, 102 SSR and six gene-based markers were polymorphic between parental lines (S1 and S2 Tables). The majority of the marker loci, 88 (81.5%), showed the expected Mendelian segregation ratio (1:2:1) for an F_2_ population whereas 20 (18.5%) marker loci, distributed across 9 chromosomes (all but chromosomes 2, 8 and 11) indicated significant segregation distortion. Among the distorted markers, 11 (55%) and 9 (45%) were biased towards MR84 and MRQ74, respectively.

### QTLs Detection and Mapping

Proline was included in our model once as an additive covariate and once as an interactive one. However, there was no interaction between the QTLs and covariate, so we only considered the model including proline as an additive covariate hereafter. Using this model, two QTLs were detected on chromosomes 4, *frg4-1*, and 8, *frg8-1* (Fig 3). We initially mapped the major QTL in the interval RM223-RM515 (2.34 cM) on the long arm of chromosome 8. This QTL, with a LOD score of 27.7, highly contributed to the phenotypic variance (49%) (Table 1). However, to saturate and resolve the region around the LOD support interval for the putative QTL, we added six polymorphic gene-based primers to this area. Consequently, the *fgr* locus was placed between RM223 (82.2 cM) and SCU015RM (83.82 cM) (Fig 3). Another important QTL was identified at RM5633, in the interval RM335-RM273, on chromosome 4. It had a LOD score of 9.3 and explained 20% of the phenotypic variation (Fig 3 and Table 1). Furthermore, a two-dimensional scan revealed no significant epistatic interactions in the entire genome of this population (Fig 4). Also, the total coverage of the linkage map was 1959.03 centiMorgans (cM), and the average marker distance was 21.73 cM (Fig 3).

**Fig 3:** Genetic map of the 12 chromosomes of a rice F_2_ population (MR84×MRQ74). Red shapes, on the linkage groups, represent QTL hotspots for the aroma trait. Chromosome numbers are indicated around the circle. The marker names and their genetic positions (cM) are shown to the right of each linkage map inside the circle. Further, LOD curve of the major QTL along with the chromosomal positions (cM) of gene-based primers are indicated on chromosome 8. Also, a red bar on this area shows the Bayesian LOD support interval.

**Fig 4:** Heat map for a two-dimensional genome scan with a two-QTL model. The maximum LOD score for the full model (two QTLs plus an interaction) is indicated in the lower right triangle. The maximum LOD score for the interaction model is indicated in the upper left triangle. A color-coded scale displays values for the interaction model (LOD threshold = 6.5) and the full model (LOD threshold = 8) on the left and right, respectively.

**Table 1:** QTLs for rice scent in the F_2_ population.

Chr.	QTL name	Nearestmarker	cM	Marker interval	NLM (cM)	NRM (cM)	LOD	AE	DE	R^2^
4	*Frg4-1*	RM5633	0.0	RM335-RM273	7.1	10.3	9.3	6.4	-2.2	20
8	*Frg8-1*	L06	0.0	RM223-SCU015RM	0.0000001	1.6	27.7	13	-2	49

cM, Genetic distance from the QTL LOD peak to the nearest marker; NLM, nearest left marker; NRM, nearest right marker; LOD, log_10_ (probability of linkage/probability of no linkage); AE, Additive effect of the allele from ‘MRQ74’ compared with that from the paternal line; DE, Dominance effect of the allele from ‘MRQ74’ compared with that from the paternal line; R^2^, Percentage of the phenotypic variance explained by each QTL.

## Discussion

In order to effectively exploit aromatic rice, a comprehensive consideration of molecular and evolutionary aspects in terms of both genomic and metabolic factors that might affect this valuable trait should be taken into account. Various studies have shown the proline is a vital precursor for 2AP biosynthesis [44, 45, 46, 47, 48]. The results presented here also confirmed a high and positive correlation between proline and fragrance (r = 0.6).

Finally, two significant QTLs were found in our population. The QTL identified on chromosome 8, with the highest effect, had a large contribution to the total phenotypic variance (Fig 3 and Table 1). The physical position of the primers tightly linked to the LOD peak of this QTL indicated that they correspond with the same locus. Based on the variants found at gene-base markers used in this research, we could also confirm the existence of a known null fragrance allele, *badh2-E7*, in MRQ74 and our mapping population. Several studies by Wanchana et al. [10], Bradbury et al. [11], and Chen et al. [12] utilizing rice genome sequence information (IRGSP 2005) have identified *badh2* as a candidate gene for fragrance on chromosome 8. Moreover, after mapping and fine-mapping, Chen et al. [12] successfully limited the *fgr* gene to a 69 kb interval. *Frg8-1* was also identified in the same area of chromosome 8 as previously reported [8, 18, 49].

QTL *frg4-1* was also detected, with minor effect, on the 4th chromosome. This locus supported previous reports of Loriex et al. [18] and Amarawathi et al. [8]. In addition to the known *BADH2* gene on chromosome 8, *BADH1*, a homolog of *BADH2* (Os04 g39020; 92% homology) [15], has been identified on chromosome 4 of rice. Based on the findings of the rice genome database for the annotated function of genes, *badh1* can be a potential candidate gene for aroma QTL *frg4-1* due to its similarity to the *badh2* gene on chromosome 8. *BADH1* is involved in stress tolerance, but its function in aroma has remained unverified [36, 50]. However, its function is similar to that of the *badh2* gene [8].

The aroma trait in this mapping population was controlled by a combination of quantitative trait loci with major and minor actions. Identifying aroma QTLs through applying such a precise method helps to further functional genomics research. Moreover, *frg4-1* and *frg8-1* can be pyramided with other favorable QTLs to obtain a substantial quality and yield enhancement in rice crop.

## Supporting Information

S1 Table Details of polymorphic SSR markers used in this research. (DOCX)

S2 Table Properties of gene-based markers. (DOCX)

S3 Table Dataset. (TXT)
